The article "Down-regulation of microRNA-138 improves immunologic function via negatively targeting p53 by regulating liver macrophage in mice with acute liver failure" was retracted in 2023. Reasons: original data or images not available; concerns about the data.

#  Down-regulation of microRNA-138 improves immunologic function via negatively targeting p53 by regulating liver macrophage in mice with acute liver failure

**DOI:** 10.1042/BSR20190763

**Published:** 2019-07-19

**Authors:** You-Qiang Wang, You-Yu Lan, Yong-Can Guo, Qin-Wei Yuan, Peng Liu

**Affiliations:** 1 Department of Laboratory Medicine, The Affiliated Traditional Chinese Medicine Hospital of Southwest Medical University, Luzhou 646000, P.R. China; 2 Department of Rheumatology and Immunology, The Affiliated Hospital of Southwest Medical University, Luzhou 646000, P.R. China; 3 Department of Hepatobiliary Diseases, The Affiliated Traditional Chinese Medicine Hospital of Southwest Medical University, Luzhou 646000, P.R. China

**Keywords:** Acute liver failure, Immune function, Macrophage, microRNA-138, P53

## Abstract

MicroRNAs (miRNAs) have been frequently identified as key mediators in almost all developmental and pathological processes, including those in the liver. The present study was conducted with aims of investigating the role of microRNA-138 (miR-138) in acute liver failure (ALF) via a mechanism involving p53 and liver macrophage in a mouse model. The ALF mouse model was established using C57BL/6 male mice via tail vein injection of Concanamycin A (Con A) solution. The relationship between miR-138 and p53 was tested. The mononuclear macrophages were infected with mimic and inhibitor of miR-138 in order to identify roles of miR-138 in p53 and levels of inflammatory factors. Reverse transcription quantitative polymerase chain reaction (RT-qPCR), Western blot analysis and ELISA were conducted in order to determine the levels of miR-138, inflammatory factors, and p53 during ALF. The results showed an increase in the levels of miR-138 and inflammatory factors in ALF mice induced by the ConA as time progressed and reached the peak at 12 h following treatment with ConA, while it was on the contrary when it came to the level of p53. Dual-luciferase reporter gene assay revealed that p53 was a target gene of miR-138. Furthermore, the results from the *in vitro* transfection experiments in primary macrophages of ALF mouse showed that miR-138 down-regulated p53 and enhanced levels of inflammatory factors; thus, improving immune function in ALF mice. In conclusion, by negatively targeting p53, the decreased miR-138 improves immunologic function by regulating liver macrophage in mouse models of ALF.

## Introduction

Liver failure is a clinical syndrome that is the final stage during the progression of liver damage due to a variety of etiological factors and is characterized by ascites, jaundice, hepatic encephalopathy, and a trend of bleeding [1]. Acute liver failure (ALF) is a serious clinical syndrome, which develops over a short period of time, associated with significant coagulopathy [2]. Drug intoxication and hepatotoxicity are the most common causes of ALF (58%), with acetaminophen overdose (46%) accounting for the majority of the cases; intracranial hypertension is the most fatal complication of ALF, which occurs in 80% of ALF patients and results in death of 25% of these patients [3]. The survival rate (spontaneous liver regeneration) of patients with ALF is 40%, but this varies significantly with the etiology of ALF [4]. The severity of acute live injury and the clinical outcome of ALF are dependent on the intensity of the uncontrolled stimulation of innate immune responses, which is a dominant factor in the pathogenesis of ALF [5]. Liver cancer, one of the malignant cancers in the world, represents a serious threat to the developing countries including China [6]. Hepatocellular carcinoma (HCC) is a prevalent disease in the liver, resulting in 70–85% liver cancer burden around the world [7]. Macrophages play a vital role in the initiation, progression, and treatment of acute liver injury [8]. Moreover, some microRNAs (miRNAs) have been found to be present in primary macrophages of mouse and human macrophage cells, including miR-146a and miR-155 [9]. Based on a previous study, macrophages with increased levels of miR-125b were found to be effective stimulators of immune responses, which is shown by the increased activation of antigen specific T cell and anti-tumor immunity [10]. Due to their effects on the various genes involved in hepatic cholesterol and lipid metabolism in the liver, miR-122 plays a major role in maintaining liver homeostasis [11].

Accumulating evidence has highlighted the role of various miRNAs in the regulation of initiation and progression of cancer as oncogenes or tumor suppressors [12]. Based on a number of studies, microRNA-138 (miR-138) has been found to be one of the most frequently down-regulated miRNAs in cancer and its down-regulation has been previously observed in a number of cancer types, including head and neck squamous cell carcinoma (HNSCC), thyroid cancer, and lung cancer [13–15]. The miR-138 targets cyclin D3 (CCND3) in HCC and cyclin D1 (CCND1) in nasopharyngeal carcinoma (NPC) [16,17]. The p53 checkpoint is known to induce the differentiation of embryonic stem cells and facilitate the suppression of self-renewal of adult stem cells like hematopoietic, neural, and mammary epithelial stem cells in somatic cells; therefore, p53 is one of the most important factors involved in tumor suppression, affecting cell differentiation, and stem cell function [18]. Current findings revealed that the overexpression of miR-21, mediated by active mTOR and Stat3 signaling, resulted in the elevation of the invasive properties to mouse keratinocytes *in vitro* and *in vivo*, while the inhibition of miR-21 in a metastatic spindle cell line resulted in the suppression of metastasis, which is originated by the loss of p53 in epithelia [19]. On the basis of the numerous findings mentioned above, we conducted the following study in order to determine the roles of miR-138 in ALF by establishing a mouse model of ALF induced by Concanamycin A (Con A) via tail vein injection, for the purpose of evaluating the dynamic expression of miR-138 in macrophages of Con A-treated mice and assessing the impact of miR-138 inhibition on the immune function of macrophages.

## Materials and methods

### Ethical statements

Animal use and experimental procedures conducted in the present study have been approved by the Experimental Animal Ethics Committee of the Affiliated Traditional Chinese Medicine Hospital of Southwest Medical University. All animal operations and experiments were compliant to the International Association for the Study of Pain (IASP) [20].

### Study subjects

C57BL/6 male mice (6–8 weeks old and weighing 18–22 g) purchased from Experimental Animal Center of Sichuan University (Chengdu, Sichuan, China) were housed under pathogen-free conditions at 22–25°C, with normal circadian rhythm, and free access to food and drinking water.

### Model establishment and pathological detection

The C57BL/6 male mice were injected with ConA via tail vein. The ConA powder purchased from Sigma-Aldrich Chemical Company (St. Louis, MO, U.S.A.) was dissolved in sterile phosphate buffer saline (PBS) to prepare a 4 mg/ml ConA solution, after which it was filtered, packaged, and stored at −20°C for further experiment. ConA solution concentration was adjusted to 20 mg/kg for the tail vein injection. According to the time of ConA treatment, the mice were assigned into normal, ConA 0 h (treatment of ConA for 0 h), ConA 1 h (treatment of ConA for 1 h), ConA 3 h (treatment of ConA for 3 h), ConA 6 h (treatment of ConA for 6 h), ConA 12 h (treatment of ConA for 12 h), and ConA 24 h (treatment of ConA for 24 h) groups. The liver tissues of each mice were obtained and fixed in 10% formalin solution (Beijing Biological Reagan, Beijing, China). Dehydration, paraffin embedding, and hematoxylin-eosin (HE) staining (Beijing Biological Reagan, Beijing, China) were carried out after 72 h. Histopathological changes of liver in mice were observed under a microscope (Olympus Corporation, Tokyo, Japan). The ConA treatment was followed by the centrifugation of 0.5 ml of whole blood from the mice in each group to obtain the serum. The levels of alanine aminotransferase (ALT) and aspartate aminotransferase (AST) (U/l) were determined by ELISA kits (eBioscience, San Diego, CA, U.S.A.) in order to verify the successful establishment of the liver failure models.

### Primary culture of liver macrophages

Following ConA treatment for 12 h, the liver macrophages in the mouse model were separated using portal vein perfusion. The mice were anesthetized with 1.5% pentobarbital sodium (Sigma-Aldrich Chemical Company, St Louis, MO, U.S.A.). The abdominal cavity was opened under a sterile condition to expose portal vein and inject perfusate (Pharmacia AB, Stockholm, Sweden). The liver tissues were treated with 0.05% collagenase (Gibco Company, Grand Island, NY, U.S.A.) and the detached liquid was filtered through a 200-mesh stainless steel net. Afterward, the liquid and the supernatant were centrifuged separately, each for 5 min. The precipitation was re-suspended with the mixture of Percoll solution and PBS (at the ratio of 9:1) and centrifuged at 715×***g*** for 20 min (Pharmacia AB, Stockholm, Sweden). The intermediate glass-like cellular layer was carefully extracted, washed, filtered through a 300-mesh stainless steel net, and centrifuged at 402×***gg*** for 10 min. The mixed cells were cultured in DMEM supplemented with 10% fetal bovine serum (FBS) for 4–6 h and rinsed 3–5 times with PBS. The cells that were found adhering to the wall were identified as the macrophages which were then cultured in DMEM containing 10% FBS at 37°C.

### Identification of primary liver macrophages

The primary liver macrophages were rinsed with PBS and detached with trypsin. The detachment was terminated with medium containing serum. Two tubes (3 × 10^5^ cells/tube) of cell suspension were prepared. One tube was added with 1 μl of phycoerythrin Cy5-conjugated anti-mouse monoclonal antibody to F4/80 (ab6640, Abcam Inc., Cambridge, MA, U.S.A.) and another tube was added with 1 μl of phycoerythrin Cy5-conjugated anti-mouse monoclonal antibody to IgG2b (ab210826, Abcam Inc., Cambridge, MA, U.S.A.) as control. After incubation for 30 min at 4°C with the avoidance of light, the excess unbound antibody was washed off with PBS containing 5% FBS. The cells were re-suspended in 500 μl of sheath solution and measured by a flow cytometer (FC500, Beckman Coulter, Inc., Chaska, MN, U.S.A.) within 1 h.

### Culture and transfection of mononuclear macrophage

The mouse mononuclear macrophage cell line RAW264.7 (ATCC, Rockville, MD, U.S.A., 1 × 10^5^ cells/well) was evenly spread throughout the culture plate; fresh and complete DMEM was used prior to transfection. The transfection mixture was prepared in accordance with the instructions on the Lipofectamine 2000 kit (Invitrogen, Carlsbad, CA, U.S.A.). Once the culture medium in the plate was absorbed, it was followed by the addition of the transfected mixture to obtain the transfected cell strain. The cells were classified into control group, ConA group [21], ConA + miR-138 mimic group, ConA + mimic negative control (NC) group, Con A + miR-138 inhibitor group, and ConA + inhibitor NC group. The nucleotide sequences used in transfection are shown in Table 1, which were synthesized by the Shanghai Zimmer Pharmaceutical Company (Shanghai, China).

**Table 1:** Nucleotide sequences

Nucleotide	Sequence
miR-138 mimic	5′- AGCUGGUGUUGUGAAUCAGGCCG-3′
Mimic-NC	5′- UUGUACUACACAAAAGUACUG-3′
miR-138 inhibitor	5′- UGGGGUAUUUGACAAACUGAUC-3′
Inhibitor-NC	5′- CAGUACUUUUGUGUAGUACAA-3′

### Dual luciferase reporter gene assay

The forecast results quoted from the Microrna.org website indicated that miR-138 targeted p53. The 3′-UTR fragment on Trp53 gene, containing the potential binding site of miR-138, was cloned into the pMIR-REPORT (Shanghai Sangon Biological Engineering Technology & Services Co., Ltd., Shanghai, China) luciferase reporter gene plasmid vector. Plasmids of the binding site of miR-138 and p53 in the wild-type (wt) and mutant (mut) loci were designed. The primer sequences of p53-3′-UTR were synthesized by the Shanghai Zimmer Pharmaceutical Company (Shanghai, China). After being sequenced, the primers were used in RAW264.7 cell transfection. The cell transfection groups were as follows: the mimic-NC group and miR-138 mimic group. According to the Lipofectamine 2000 (Invitrogen Inc., Carlsbad, CA, U.S.A.) kit, the cells were co-transfected with 200 ng of pMIR-REPORT-p53 3′UTR or pMIR-REPORT-mut-p53 3′UTR and 30 nM of miR-138 mimic or NC for 24 h at 37°C. Fluorescence intensity was tested according to the Dual-Luciferase Reporter Gene Detection System (Promega Corporation, Madison, WI, U.S.A.).

### Reverse transcription quantitative polymerase chain reaction (RT-qPCR)

Total RNA was extracted from cells using Trizol (Invitrogen, Carlsbad, CA, U.S.A.). The extracted RNA was reverse transcribed using the PrimeScript® RT reagent kit by NanoDrop2000 (Thermo Fisher Scientific, San Jose, CA, U.S.A.). The specific primers were required in reverse transcription of miR-138 and U6. The reverse transcription primer sequences were as follows: U6: 5′-GTCGTATCCAGTGGCAGGGTCCGAGGTATTCGCACTGGATACGACAAAAATA-3′; miR-138: 5′-CTCAACTGGTGTCGTGGAGTCGGCAATTCAGACACTTAG-3′. PCR primers were designed in accordance with the gene sequences published in the Genebank database using Primer 5.0 Primer Design Software (Table 2). The primers were synthesized by Shanghai Sangon Biological Engineering Technology & Services Co., Ltd. (Shanghai, China). The reaction solution was configured and the reaction conditions were set according to the instructions of reverse transcription quantitative polymerase chain reaction (RT-qPCR) kit. The ABI PRISM 7500 real-time PCR System (ABI Company, Oyster Bay, NY, U.S.A.) and SYBR Green I Fluorescent Kit (Takara Biotechnology Ltd., Dalian, Liaoning, China) were applied with U6/β-actin as the internal reference. The reliability of the PCR result was evaluated by the solubility curve and the *C*_T_ value was obtained using the following formula: △*C*_t_ = *C*_T_ (target gene) – *C*_T_ (reference), △△*C*_t_ = △*C*_t_ (experimental group) – △*C*_t_ (control group). The relative level of target gene was calculated using 2^−△△*C*^_t_ [22].

**Table 2:** Primer sequence for RT-qPCR

Genes	Forward primer (5′-3′)	Reverse primer (5′-3′)
miR-138	GGTGTCGTGGAGTCGGCAA	AACTTCACAACACCAGCTTA
U6	CTCGCTTCGGCAGCACA	AACGCTTCACGAATTTGCGT
p53	CCAGGATGTTGCAGAGTTGTTA	CTCACGACCTCAGTCATGTGTT
TNF-α	CAACGCCCTCCTGGCCAACG	TCGGGGCAGCCTTGTCCCTT
IL-1β	AGAGCATCCAGCTTCAAATCTC	CAGTTGTCTAATGGGAACGTCA
IL-6	TAGTCCTTCCTACCCCAATTTCC	TTGGTCCTTAGCCACTCCTTC
β-actin	AGTGTGACGTTGACATCCGT	GCAGCTCAGTAACAGTCCGC

Abbreviations: TNF, tumor necrosis factor; IL, interleukin.

### Western blot analysis

The total protein was extracted from the cells, and the protein concentration was detected according to the instructions of the Bicinchoninic Acid (BCA) Kit (Wuhan Boster Biological Technology Ltd., Wuhan, Hubei, China). The protein samples were then added to the sample buffer and boiled at 95°C for 10 min. The samples were loaded at 30 μg/well and separated by 10% PAGE. The electrophoretic voltages were 80 V (spacer gel) and 120 V (separation gel). Afterward, the samples were transferred onto a polyvinylidene fluoride (PVDF) membrane by the wet transfer method with constant current of 100 mv for 50–90 min. The membrane was blocked with 5% bovine serum albumin (BSA) at room temperature for 1 h, and then incubated with the primary antibodies, mouse monoclonal antibody to p53 (1:1000; ab26, Abcam Inc., Cambridge, MA, U.S.A.), mouse monoclonal antibody to p-p53 (1:1000; 9284, CST, Beverly, MA, U.S.A.), and mouse monoclonal antibody to β-actin (1:1000; ab8226, Abcam Inc., Cambridge, MA, U.S.A.) at 4°C overnight. After being rinsed 3 times with tris-buffered saline with tween (TBST) (5 min/time), the membrane was added with secondary antibody, goat anti-mouse antibody (1:2000; ab6789, Abcam Inc., Cambridge, MA, U.S.A.) for incubation at room temperature for 1 h, and then rinsed 3 times with TBST (5 min/time). The chemiluminescent reagent was used for development and β-actin was used as an internal reference. The gray value target band was analyzed using the Image J software.

### Enzyme-linked immunosorbent assay (ELISA)

The total protein was extracted from the cells. ELISA assay was performed with strict accordance with the instructions of the ELISA kit (eBioscience, San Diego, CA, U.S.A.). The ELISA kit was equilibrated at room temperature for 20 min and the washing solution was prepared. Following dissolution, 100 μl of standard sample was added to the reaction plate for the standard curve plotting. Based on the protein concentration determined by the BCA kit, the samples were diluted for further detection (diluted for 2 times), followed by the addition of 100 μl of samples to the reaction wells for incubation at 37°C for 90 min, which were then washed 3 times. Afterward, 100 μl of freshly prepared biotinylated antibody working solution was added for incubation at 37°C for 60 min and washed 3 times. Subsequently, 100 μl of freshly prepared enzyme-binding reactants working solution was added for incubation at 37°C for 30 min. The plate was washed 3 times and 100 μl of substrate was added to each well. The mixture was gently shaken and incubated, avoiding exposure to light at 37°C for 15 min. Stop buffer (100 μl) was added to each well in a quick manner to terminate the reaction, and the microplate reader (BioTek Instruments, Inc., Vermont, U.S.A.) was applied to test the optical density (OD) value of each wells within 3 min. According to the OD value, the standard curve was plotted and analyzed based on tumor necrosis factor-α (TNF-α), interleukin (IL)-6, and IL-1β content.

### Statistical analysis

The data were analyzed by SPSS 18.0 Statistical Software (IBM Corp., Armonk, NY, U.S.A.). The measurement data were expressed as mean ± standard deviation. The *t* test was conducted to compare data obeying the normal distribution between two groups. The comparison among multi-groups was performed by one-way analysis of variance. Enumeration data were expressed as percentages and rates and analyzed using chi-square test. A *P*<0.05 was indicative of statistical significance.

## Results

### ALF mouse models were established successfully

HE staining was used identify the pathological characteristics of ALF in mice, and the findings revealed that in comparison with the control group, there were no significant changes in liver pathology in the ConA 0 h group; the ConA 1 h group exhibited only small dispersed polymorphonuclear leukocytes infiltration and rare necrotic foci; small and scattered inflammatory necrosis with polymorphonuclear leukocyte infiltration was found in the ConA 3–6 h group; there was obvious patchy necrosis and portal congestion and coagulation phenomenon in the ConA 12–24 h group (Figure 1A). All of the aforementioned findings indicated that ConA induced ALF in mice, and the degree of ALF increased in severity as time progressed. Figure 1B showed that liver failure was observed in mice treated with ConA for 6–24 h with significantly increased ALT and AST levels. The above results showed the successful establishment of ConA-induced liver failure models.

**Figure 1:** ConA induced ALF in mouse HE staining images of liver tissues of mice in each group (yellow arrows indicate necrotic inflammatory cells) (400×) (**A**). The serum ALT and AST levels of mice in each group (**B**). The control group: liver tissues without treatment. The ConA treatment groups were tissue-stained after their processing time. *n*=6. *P<0.05 vs the control group. ConA, Concanamycin A

### Primary mouse liver macrophages are identified

Subsequently, the liver tissues of ALF mice induced by ConA and normal mice were separated to obtain macrophages. F4/80 staining labeled by phocoerythrin (PE)-Cy5 was identified by flow cytometry. F4/80 is a characteristic surface marker of mouse mature macrophages. Flow cytometry results showed that the purity of liver macrophages in the ConA 12 h group was 94.8%, while that in the control group was 95.2% (Figure 2A–D), indicating that the isolated cells were liver macrophages.

**Figure 2:** The primary liver macrophages were identified in mice Positive liver macrophage ratio labeled by IgG2b after mice were treated with ConA for 12 h determined by flow cytometry (**A**). The positive liver macrophage ratio labeled by F4/80 after mice were treated with ConA for 12 h by flow cytometry (**B**). The positive liver macrophage ratio labeled by IgG2b in mice of the control group by flow cytometry (**C**). The positive liver macrophage ratio labeled by F4/80 in mice of the control group by flow cytometry (**D**). *n*=3. ConA, Concanamycin A.

### Levels of miR-138 and inflammatory factors increase, while level of p53 decreases during ALF

Next, RT-qPCR (Figure 3A–E), Western blot analysis (Figure 4A,B), and ELISA (Figure 5A–C) were performed for measurement of miR-138, TNF-α, IL-6 and IL-1β, and p53 levels as well as the extent of p53 phosphorylation during ALF. RNA was extracted from primary liver macrophages of ALF mice induced by ConA. Based on the results, there were no significant changes observed in the ConA 0 h group compared with the control group. The level of miR-138 and levels of inflammatory factors (TNF-α, IL-6, and IL-1β) increased as time progressed, which reached its peak in the ConA 12 h group, but significantly decreased in the ConA 24 h group as compared with those in the ConA 12 h group (all *P*<0.05). The mRNA and protein levels of p53 showed the opposite trend of miR-138. Besides, the extent of p53 phosphorylation was gradually elevated following the treatment of ConA. The aforementioned findings revealed that the increased levels of miR-138 and inflammatory factors, together with lower levels in p53 were associated with ALF.

**Figure 3:** miR-138 expression and mRNA levels of TNF-α, IL-6, and IL-1β were increased, while mRNA level of p53 was decreased in liver macrophages The miR-138 level in response to ConA 0 h, ConA 1 h, ConA 3 h, ConA 6 h, ConA 12 h, ConA 24 h (**A**). The mRNA level of p53 in response to ConA 0 h, ConA 1 h, ConA 3 h, ConA 6 h, ConA 12 h, ConA 24 h (**B**). The mRNA level of TNF-α in response to ConA 0 h, ConA 1 h, ConA 3 h, ConA 6 h, ConA 12 h, ConA 24 h (**C**). The mRNA level of IL-6 in response to ConA 0 h, ConA 1 h, ConA 3 h, ConA 6 h, ConA 12 h, ConA 24 h (**D**). The mRNA level of IL-1β in response to ConA 0 h, ConA 1 h, ConA 3 h, ConA 6 h, ConA 12 h, ConA 24 h (**E**). The ConA treatment groups were cell-treated after their processing time. *P<0.05 vs the control group. ^#^*P*<0.05 vs the ConA 12 h group. *n*=6. One-way analysis of variance was used for multi-group comparisons followed by Tukey’s *post hoc* test.ConA, Concanamycin A.

**Figure 4:** Protein levels of p53 were reduced following treatment of ConA The protein level of p53 and the extent of p53 phosphorylation in primary macrophages of ALF mice (**A**). The gray value of p53 protein bands (**B**). The ConA treatment groups were cells treated after their processing time. *P<0.05 vs the control group. ^#^*P*<0.05 vs the ConA 12 h group. *n*=6. One-way analysis of variance was used for multi-group comparisons followed by Tukey’s *post hoc* test. ConA, Concanamycin A.

**Figure 5:** Protein level of p53 after ConA treatment in ALF mice Increased levels of TNF-α (**C**), IL-6 (**B**), and IL-1β (**A**) after treatment of ConA. The ConA treatment groups were cells treated after their processing time. *P<0.05 vs the control group. ^#^*P*<0.05 vs the ConA 12 h group. *n*=6. One-way analysis of variance was used for multi-group comparisons followed by Tukey’s *post hoc* test. ConA, Concanamycin A.

### miR-138 targets p53

The p53 is an important regulator in the process of cell apoptosis. It plays an important role in cell senescence in most murine tissues. The deletion of p53 promotes the development of liver fibrosis and tumor progression. Based on the findings from the online analysis website (microrna.org), miR-138 targets p53 (Figure 6A). There was a significant inhibition in the luciferase activity of p53-wt 3′UTR by miR-138 compared with that of the NC group (*P*<0.05), but the luciferase activity of p53-mut 3′UTR was not changed (*P*<0.05). This indicated that miR-138 targeted p53 (Figure 6B). Pearson correlation analysis showed a negative correlation (*r*=-0.948, *P*<0.001) between the RT-qPCR results of miR-138 and p53 (Figure 6C). The results showed that p53 was a target gene of miR-138.

**Figure 6:** miR-138 targets p53 The binding sites of miR-138 and p53-3′UTR predicted by public databases (**A**). The dual-luciferase reporter assay for confirmation of the targeting relationship between miR-138 and p53 (**B**). Pearson’s analysis of the relationship between miR-138 and p53 (the data from panel 3A and B) (**C**). *P<0.05 vs the NC group. The experiment was repeated 3 times. The cells in each group were detected 24 h after transfection. *t* test was used in comparisons between two groups. ConA, Concanamycin A.

### Downregulated miR-138 improves immune function of ALF in mice by down-regulating p53 and enhancing levels of inflammatory factors

Finally, RT-qPCR, Western blot analysis, and ELISA were applied in order to identify the levels of miR-138, p53, TNF-α, IL-6, and IL-1β by determining the levels of RNA in RAW264.7 cells (Figures 7A–E and 8A–E). Compared with the control group, the ConA and miR-138 mimic groups exhibited significant increase of miR-138 level (both *P*<0.05). Compared with the ConA + miR-138 group, there was a significant inhibition in miR-138 level in the the ConA + miR-138 inhibitor group (*P<0.05*). The mRNA and protein levels of p53 significantly decreased in the ConA and miR-138 mimic groups (both *P<0.05*), while they were increased in the ConA + miR-138 inhibitor group (*P<0.05*). The mRNA and protein levels of IL-6, TNF-α, and IL-1β significantly increased in the ConA + miR-138 mimic group (all *P<0.05*), while they remarkably decreased in the ConA + miR-138 inhibitor group (all *P<0.05*). These findings indicated that miR-138 inhibited the level of p53 and promoted the level of inflammatory factors; thus, promoting the improvement of immune function and protection from ALF.

**Figure 7:** Elevated mRNA levels of TNF-α, IL-6, and IL-1β and reduced level of p53 after infection of miR-138 inhibitor in RAW264.7 cells The miR-138 level of cells treated with ConA alone and with miR-138 mimic or inhibitor (**A**). The mRNA level of p53 of cells treated with ConA alone and with miR-138 mimic or inhibitor (**B**). The mRNA level of IL-6 of cells treated with ConA alone and with miR-138 mimic or inhibitor (**C**). The mRNA level of TNF-α of cells treated with ConA alone and with miR-138 mimic or inhibitor (**D**). The mRNA level of IL-1β of cells treated with ConA alone and with miR-138 mimic or inhibitor (**E**). *P<0.05 vs the control group; ^#^*P*<0.05 vs the ConA group. The experiment was repeated 3 times. The cells in each group were detected 24 h after transfection. One-way analysis of variance was used for multi-group comparisons followed by Tukey’s *post hoc* test. ConA, Concanamycin A.

**Figure 8:** Protein level of p53 was decreased by miR-138 The p53 protein level in cells among the six groups (**A**). The gray value of p53 protein bands using the Image J software (**B**). The TNF-α protein level in cells among the six groups (**C**). The IL-6 protein level in cells among the six groups (**D**). The IL-1β protein level in cells among the six groups (**E**). *P<0.05 vs the control group. ^#^*P*<0.05 vs the ConA group. The experiment was repeated 3 times. The cells in each group were detected 24 h after transfection. One-way analysis of variance was used for multi-group comparisons followed by Tukey’s *post hoc* test. ConA, Concanamycin A.

## Discussion

ALF is a serious condition that leads to the deterioration of liver function in patients with previously well-functioning liver and is often accompanied by coagulopathy, progressive hepatic encephalopathy, and jaundice, and could potentially result in multiple organ dysfunction or failure [23]. Non-coding RNAs (ncRNAs) including lncRNAs and miRNAs are critical regulators of numerous cellular processes, and are involved in the development of cancers. ncRNAs could regulate the expression of transcription factors, mediate the recombination and modification of chromatin, and reduce the regulation of mRNA transcription on gene expression. ncRNAs are essential for intracellular homeostasis and are widely known to participate in the regulation of inflammation [24,25]. miR-138 has various functions and there has been a growing interest in this molecule due to its down-regulation that has been observed during carcinogenesis [26]. The present study highlights the effects of miR-138 on the immune function of mice with ALF, and the findings were highly suggestive of the concept that the negative regulation of p53 by downregulated miR-138 could affect the function of liver macrophages and enhance the immune function of mice with ALF.

Initially, our findings revealed that there was an increase in the levels of miR-138, which was proportional with the time of ConA induction, which reached its peak at 12 h following treatment with ConA, but decreased after treatment with ConA for 24 h. miR-138 has been reported to have multiple biological functions, and is often down-regulated in human cancers [26,27]. A previous study found that a significant overexpression in miR-138 results in the inhibition of hypoxia-induced apoptosis of cardiomyocyte by decreasing the level of pro-apoptotic protein-2 (Lcn2), which was consistent with our findings [28]. In addition, the frequent down-regulation of miR-138 may modulate CCND3 and act as a tumor suppressor in HCC, serving as an effective therapeutic agent in miRNA-based HCC treatment [29]. In addition, we found that p53 level reduced gradually with the time of ConA induction. p53 is widely expressed in a variety of tissues at a low level, and significant up-regulation of p53 has been linked with the presence of tumor tissues and inflamed/damaged tissues [30,31]. It is known that cells would activate their signaling pathway and the relevant factors to induce gene transcription; thus, adapting to the changes of the external conditions. However, p53 is a critical molecule activated by cells under the stimulation of genotoxicity and non-genetic toxicity and its activation could activate different types of target genes, induce cellular changes including cell arrest, apoptosis, and necrosis, and participate in DNA damage repair [32]. Intracellular regulation of p53 is mainly achieved by transcription and modification. When cells are exposed to DNA damage, hypoxia, or high temperature, the MDM2-catalyzed ubiquitin proteasome-dependent degradation signaling pathway is inhibited, leading to p53 degradation, reduced p53 transfer from nucleus, and p53 aggregation in nucleus, and eventually producing cellular response to physiological stress [33]. It was shown that the activation of p53 is affected by cell type, stimulation form, and cellular environment [34,35]. It means that p53 activates the downstream target genes of different genomes in response to different stimulation signals [36,37]. Therefore, ConA treatment affects the expression of downstream genes and other cell signal proteins regulated by p53. p53 has also been found to interact with NF-κB, and their activities are negatively associated [38]. It has been reported that p53 deficiency resulted in the remarkable increase in the occurrence of autoimmune diabetes in mouse, which might be due to the suppression of pro-inflammatory cytokines and STAT-1 [30]. Dual luciferase reporter gene assay showed that miR-138 targeted p53. It has been reported that miR-138 may regulate p53 in clinical studies, including femoral head necrosis, fibromatosis, and lung cancer [39–42]. It has been noted that miR-138 is also involved in the regulation of p53 in mice and rat cells, but this was not the case in non-small cell lung cancer cells in humans [43]. This finding highly suggests that there might be a species-specific difference between the regulation of miRNA on its target and the regulation of miRNA by other proteins. miR-138 regulates the signal transduction of p53 to induce inflammation. It was revealed that miR-138 could directly target the 3′UTR of p53 to down-regulate the expression of p53 and the downstream genes; additionally, the aberrantly expressed p53 with a mut 3′UTR cannot be targeted by miR-138 and could severely damage the role of miR-138 in p53 signaling; thus, leading to the induction of inflammation [44,45].

Subsequently, it was revealed that the levels of inflammatory factors (IL-6, TNF-α, and IL-1β) were increased with the time of ConA induction and reached the peak at 12 h after treatment with ConA, but decreased after treatment with ConA for 24 h. A recent study identified the release of inflammatory cytokines as the key mediators involved in the pathogenesis of ConA-induced hepatitis [46]. Moreover, the production of IL-6, TNF-α, and IL-1β was found to have a strong inhibitory effect on methylprednisolone (MP) using monocytes within the first 18 h for fusion following stimulation [47]. Furthermore, the results of *in vitro* transfection experiments, in primary macrophages of ALF mice and RAW264.7 cells, were consistent with the results of primary hepatic macrophages in mice. It has also been demonstrated that miR-138 could inhibit the level of p53 and promote the level of inflammatory factors. Zhang *et al.* proved that the decline of p53 in synovial fibroblasts promotes the activation of the NF-κB and MAPK signaling pathways, which resulted in the elevation of IL-6 secretion [48].

## Conclusion

The key findings from the present study revealed that an ALF mouse model can provide a remarkable insight into ConA-induced ALF in mice and the use of this mouse model was the key in determining the essential mechanism by which downregulated miR-138 affects the function of liver macrophages and enhances the immune function of mice with ALF by negatively targeting p53. ConA-induced hepatitis is an ideal animal model for the pathophysiology of human autoimmune hepatitis, and has been widely used to elucidate a variety of human T-cell-mediated liver disease [46]. There’s been numerous evidences suggesting that the apoptotic signaling pathways are activated by IFN-γ/STAT1 in ConA-induced T cell hepatitis [49]. miR-138 was also found to closely correlated with the PI3K/AKT signaling pathway [50], which participates in d-galactosamine/lipopolysaccharide-induced ALF [51]. Although the study highlighted the aforementioned key points, it was not able to verify the binding relationship between miR-138 and p53 *in vivo*. Therefore, further studies are required in order to explore the underlying mechanism of miR-138 in regulating immune function in mice with ALF and other pathways associated with miR-138 for further verification of the conclusion from our study.

## Abbreviations

ALF: acute liver failure
ALT: alanine aminotransferase
AST: aspartate aminotransferase
BCA: bicinchoninic acid
CCND3: cyclin D3
Con A: concanamycin A
FBS: fetal bovine serum
HCC: hepatocellular carcinoma
HE: hematoxylin-eosin
IL: interlukin
MAPK: mitogen-activated protein kinase
miR-138: microRNA-138
miRNAs: microRNAs
mut: mutant
NC: negative control
ncRNA: non-coding RNA
OD: optical density
PBS: phosphate buffer saline
PE: phycoerythrin
PI3K: phosphatidylinostitol 3-kinase
RT-qPCR: reverse transcription quantitative polymerase chain reaction
STAT3: signal transducer and activator of transcription-3
TBST: tris-buffered saline with tween
TNF: tumor necrosis factor
wt: wild-type
